This article has been retracted.

# Adropin Inhibits Vascular Smooth Muscle Cell Osteogenic Differentiation to Alleviate Vascular Calcification via the JAK2/STAT3 Signaling Pathway

**DOI:** 10.1155/2022/9122264

**Published:** 2022-07-27

**Authors:** Li Wang, Fulu Jin, Peiyu Wang, Shiqiang Hou, Tao Jin, Xiansong Chang, Liangping Zhao

**Affiliations:** ^1^Department of Cardiology, The Second Affiliated Hospital of Soochow University, Suzhou, Jiangsu, China 215004; ^2^Emergency Department, The Second Affiliated Hospital of Soochow University, Suzhou, Jiangsu, China 215004; ^3^Department of Cardiology, Shanghai Institute of Cardiovascular Disease, Zhongshan Hospital, Fudan University, Shanghai, China 200032

## Abstract

Vascular calcification is characterized as the deposition of hydroxyapatite mineral in the form of calcium-phosphate complexes in the vasculature. Transdifferentiation between vascular smooth muscle cells (VSMCs) and osteoblast-like cells is considered essential in the progression of vascular calcification. The pathophysiological mechanisms underlying vascular calcification and VSMC osteogenic differentiation remain to be fully elucidated, and the development of novel therapies is required. In the present study, PCR and western blot analysis were conducted to quantify the mRNA and protein expression levels of calcification-associated markers (bone morphogenetic protein 2, alkaline phosphatase, osteoprotegerin, osteocalcin, and runt-related transcription factor 2) and adropin in VSMCs and rat vascular tissues. The calcification of VSMCs was assessed using alizarin red staining. Moreover, adropin expression levels in VSMCs were analyzed using immunofluorescence. Lentiviral transfection and small interfering RNA were used for overexpression and knockdown of adropin in VSMCs, respectively. The results demonstrated that adropin alleviated vascular calcification in vivo. Moreover, adropin also inhibited osteogenic differentiation and the calcification of VSMCs in vitro. Notably, results of the present study revealed that the tyrosine protein kinase JAK2 (JAK2)/signal transducer and activator of transcription 3 (STAT3) signaling pathway played a key role in the aforementioned inhibition. In conclusion, the results of the present study demonstrated that adropin inhibited VSMC osteogenic differentiation to alleviate vascular calcification via the JAK2/STAT3 signaling pathway.

## 1. Introduction

Vascular calcification is defined as the deposition of calcium phosphate mineral in the cardiovascular system, mainly in blood vessels, myocardium, and cardiac valves [1]. Pathologic calcification of vascular calcification may decrease the elasticity of blood vessels and elevate blood pressure, which is one of the most important factors determining patients' morbidity and mortality worldwide [2]. The transdifferentiation of vascular smooth muscle cells (VSMCs) into osteoblast-like cells has previously been recognized as a key event in the progression of vascular calcification [3, 4]. Therefore, it is important to identify novel targets to alleviate VSMC transdifferentiation, in order to improve the treatment options for vascular calcification.

Adropin is a highly conserved peptide hormone (length, 76 amino acids), which is mainly secreted from the liver. Results of a previous study demonstrated that adropin may play a key role in the regulation of the vascular endothelium [5]. Moreover, results of further studies have suggested that adropin is an important regulatory component in cardiovascular functions and exerts a protective effect on the pathogenesis and development of certain cardiovascular diseases [6, 7]. Thapa et al. demonstrated that adropin treatment may recover the glucose oxidation of the heart in prediabetic obese mice [8]. However, few studies have reported the influence of adropin on the pathogenesis of vascular calcification.

Protein kinase JAK2 (JAK2) is an upstream kinase in the signal transducer and activator of transcription 3 (STAT3) phosphorylation pathways [9]. Lu et al. demonstrated that adiponectin may inhibit *β*-glycerophosphate-induced VSMC calcification via JAK2/STAT3 signaling [10]. He et al. also demonstrated that the JAK2/STAT3/bone morphogenetic protein 2 (BMP2) axis is associated with erythropoietin-related calcification in rat VSMCs [11]. These studies demonstrated that the JAK2/STAT3 signaling pathway may play a role in the progression of VSMC calcification. Based on the aforementioned experiments, the present study is aimed at investigating whether the JAK2/STAT3 axis played a role in the process of adropin-mediated vascular calcific protection, both in vivo and in vitro.

In the present study, we hypothesized that adropin treatment may exert a positive effect in the treatment of vascular calcification and the JAK2/STAT3 signaling pathway may be involved. The inhibitory impact of adropin on vascular calcification was investigated in an animal model and in osteogenic differentiated VSMCs in the present study. The findings of the present study may provide a novel theoretical basis for further understanding the molecular mechanisms associated with the protective effects of adropin in vascular calcification. They may help us to develop new methods and medicine based on adropin and JAK2/STAT3 signaling to treat vascular calcification diseases, such as atherosclerotic disease, hypertension, diabetes, and chronic kidney diseases.

## 2. Materials and Methods

### 2.1. Cell Culture

The human VSMC line was obtained from The Cell Bank of Type Culture Collection of The Chinese Academy of Sciences. 1640 medium (Hyclone; Cytiva) supplemented with 20% fetal bovine serum (FBS; Gibco; Thermo Fisher Scientific, Inc.) was used to culture VSMCs. VSMCs were seeded into T-75 flasks and incubated in a humidified incubator supplied with 5% CO_2_ at 37°C. The medium was changed every 2 days.

Osteogenic differentiation medium (DMEM supplemented with 1 M *β*-Glycerophosphate and 1 M CaCl_2_) was used for osteogenic differentiation in VSMCs. VSMCs were cultured in osteogenic differentiation medium for 8-10 days to obtain an osteoblast-like phenotype. The culture medium was changed every day.

### 2.2. Immunofluorescence

QuickBlock™ immunostaining blocking reagent (Beyotime Institute of Biotechnology) was used to block nonspecific binding sites, and 3% H_2_O_2_ was used to block endogenous peroxidase. Subsequently, the plates were incubated with the primary antibody overnight at 4°C. After washing to remove the primary antibodies, the plates were incubated with a secondary antibody for 2 h at room temperature. A laser confocal microscope (Zeiss AG) was used to visualize target proteins. The primary and secondary antibodies used are listed in Supplementary Table S1.

### 2.3. Alizarin Red Staining

Alizarin red staining was performed using the Alizarin Red Staining kit (Wuhan Servicebio Technology, Co., Ltd.) to determine the extent of matrix calcification. The protocol was performed in accordance with the manufacturer's instructions. Briefly, cultured VSMCs were fixed with 4% paraformaldehyde. A total of 1 ml staining reagent was added to every well of a 6-well plate for 60 min. Subsequently, the staining reagent was washed off using ice-cold PBS. All images were captured using an optical microscope (Zeiss AG), and all results are presented as the relative integrated optical density IOD (sum/area sum).

### 2.4. Alkaline Phosphatase (ALP) Activity Assay

ALP activity was measured using an ALP Color Development kit (Beyotime Institute of Biotechnology). Briefly, VSMCs were incubated with ALP-labeled antibodies and washed 3-5 times for 4-6 min each time. Subsequently, each solution was washed off. Following the last wash, a BCIP/nitrotetrazolium chloride blue (NBT) dye working solution was added, and the sample was incubated at room temperature for 30 min. All results are presented as the relative IOD (sum/area sum).

### 2.5. Western Blotting

Radioimmunoprecipitation assay (RIPA) buffer (Sigma-Aldrich; Merck KGaA) was used to extract proteins from VSMCs or rat vascular tissues. The amount and quality of the protein were checked by bicinchoninic acid assay (BCA) (Beyotime, China) in a Synergy H1 Microplate Reader (BioTek, USA). Diluted protein was incubated for 5 min at 100°C, and then equal amounts of protein were loaded on a 12% gel from a TGX Stain-Free FastCast Acrylamide Kit (Bio-Rad, USA) and finally transferred onto a 0.45 *μ*m PVDF membrane (GE Healthcare, USA). Subsequently, specific primary antibodies were used for overnight incubation at 4°C. The following day, the membranes were washed 3-5 times and incubated with the secondary antibodies at room temperature for 1.5 h. Proteins were visualized using chemiluminescence reagents (Absin, China). Band intensities were quantified using Image-Pro Plus 6.0 (Media Cybernetics, USA), and GAPDH was used for normalization. The primary antibodies and secondary antibodies used for western blot analysis are detailed in Supplementary Table S1.

### 2.6. Reverse Transcription-Quantitative (RT-q) PCR

Briefly, total RNA from VSMCs or rat vascular tissues was extracted using an DNA/RNA/Protein Extract kit (Thermo Fisher Scientific, Inc.), and cDNA was synthesized using a reverse-transcribed kit (Shanghai Yeasen Biotechnology, Co., Ltd.) on a Mastercycler X50 (Eppendorf). Then, qPCR was performed using ChamQ SYBR Color qPCR Master Mix (Vazyme) in a ViiA 7 system (Life Technologies, USA). The relative expression levels of target genes were calculated using the 2^-*ΔΔ*CT^ method, and GAPDH was used for normalization. The primers used for RT-qPCR are listed in Supplementary Table S2.

### 2.7. Small Interfering (si) RNA

To inhibit the adropin expression, cultured VSMCs at 70-80% confluency were transfected with a specific siRNA (100 nM) or scrambled siRNA (100 nM) using Lipofectamine® 3000 (Invitrogen; Thermo Fisher Scientific, Inc.). Genomeditech (Shanghai, China) assisted in the design and production of siRNA. Following incubation at 37°C with 5% CO_2_ for 6 h, the medium was replaced with DMEM (Hyclone; Cytiva) containing 10% FBS (Gibco; Thermo Fisher Scientific, Inc.). Following transfection, the cells were harvested after 48 h for RNA extraction.

### 2.8. Lentiviral Transfection

The adropin overexpression was carried out using a lentiviral vector. Negative control vectors and adropin lentiviral vectors were synthesized by GeneChem, Inc. Briefly, VSMCs were cultured into 6-well plates and transfected with the lentivirus vector using Lipofectamine® 3000 (Invitrogen; Thermo Fisher Scientific, Inc.) according to the manufacturer's instructions. The medium was changed every 6 h, and VSMCs were cultured for 72 h at 37°C.

### 2.9. Animal Experiments

SD rats (male; body weight, 180-200 g) were obtained from the Shanghai Model Organisms Center. All rats were housed in an environment with a temperature of 23 ± 1°C, a humidity of 50 ± 10%, and a light/dark cycle of 12/12 h. Rats were given access to standard rat food and water ad libitum. Animal handling and treatment were performed in compliance with Chinese national guidelines. Ethical approval for all experimental protocols was issued by the Animal Care Committee of The Second Affiliated Hospital of Soochow University (ethics approval No. SUDA20200226A01).

To establish the vascular calcification model, rats were injected with vitamin D3 (300,000 IU/kg) and simultaneously administrated with nicotine (25 mg/kg in 3 ml peanut oil) at 9 : 00 a.m. on the first day. The nicotine administration was repeated at 5 : 00 p.m. on the same day, and the modeling continued for 8 weeks. Rats in the control group received an injection of saline and oral gavage of peanut oil. Rats in the adropin group were administered 50 mg/kg adropin intragastrically (Thermo Fisher Scientific, Inc.) each day. After 8 weeks of treatment, all rats were injected with ketamine (75 mg/kg; i.p.)/medetomidine (0.5 mg/kg; i.p.) and euthanized by cervical dislocation. The vascular tissues were collected for subsequent analyses.

### 2.10. Statistical Analysis

Statistical analysis was performed using SPSS 21.0 Software (IBM Corp.). One-way ANOVA followed by a Bonferroni post hoc test was performed to examine the quantitative data. Data are presented as the mean ± standard deviation. *p* < 0.05 was considered to indicate a statistically significant difference.

## 3. Results

### 3.1. Adropin Is Expressed at Low Levels in Calcific Vascular Tissues and VSMCs Undergoing Osteogenic Differentiation

The expression levels of adropin were analyzed in the progression of vascular calcification. A C57/BL6 rat model was developed with vascular calcification for in vivo investigation, and VSMCs were stimulated for osteogenic differentiation for in vivo investigation. As shown in Figures 1(a) and 1(b), compared with the control and vehicle groups, the protein levels of adropin were significantly decreased in calcific vascular tissues and osteogenic differentiated VSMCs. Moreover, the mRNA levels of adropin in osteogenic differentiated VSMCs were also reduced (Figure 1(c)). These results were further verified using immunofluorescence (Figures 1(d) and 1(e)). Collectively, the results of the present study demonstrated that adropin is expressed at low levels in calcific vascular tissues and osteogenic differentiated VSMCs.

### 3.2. Adropin Inhibits VSMC Osteogenic Differentiation In Vitro

As adropin was expressed at low levels in osteogenic differentiated VSMCs, the impact of adropin in the calcification of VSMCs was subsequently explored. Adropin was silenced using siRNA and overexpressed using plasmid transfection in VSMCs (Figures 2(a) and 2(b)). Subsequently, the expression levels of calcification-associated markers, namely, BMP2, ALP, osteoprotegerin (OPG), osteocalcin (OCN), and runt-related transcription factor 2 (Runx2), were determined in each group of VSMCs. Compared with osteogenic differentiated VSMCs, results of the western blotting analysis demonstrated that the protein expression levels of calcification markers were significantly increased in si-adropin transfected VSMCs in osteogenic medium (Figures 3(a) and 3(b)). Furthermore, the expression of these calcification markers was decreased following the adropin overexpression in VSMCs in osteogenic medium. Thus, the results of the present study suggested that adropin may inhibit VSMC osteogenic differentiation in vitro.

### 3.3. Adropin Inhibits JAK2/STAT3 Activation in Osteogenic Differentiated VSMCs In Vitro

As the JAK2/STAT3 signaling pathway may regulate VSMC calcification in vitro [10, 11], whether adropin also inhibited the activation of JAK2/STAT3 to alleviate calcification in VSMCs was further investigated. As shown in Figures 2(a) and 2(c), comparing with normal VSMCs, the activation of JAK2/STAT3 was increased in si-adropin transfected VSMCs. In addition, the overexpression of adropin neutralized the promoting effect of osteogenic medium in VSMCs. In conclusion, these findings indicated that adropin may inhibit JAK2/STAT3 signal activation in osteogenic differentiated VSMCs in vitro.

### 3.4. Adropin Inhibits VSMC Calcification In Vitro

The calcification of VSMCs was visualized using alizarin red staining. Compared with the control group, the alizarin red positive area was significantly increased in osteogenic differentiated VSMCs and VSMCs with adropin expression knocked down (Figure 4(a)). However, the overexpression of adropin neutralized the promoting impact of alizarin red staining in VSMCs. Moreover, a calcium ion assay was carried out to evaluate the content of calcium in VSMCs. As shown in Figure 4(b), following the adropin overexpression in VSMCs in osteogenic medium, calcium levels were significantly reduced. The mRNA expression levels of calcification-associated markers (BMP2, ALP, OPG, OCN, and Runx2) in VSMCs also confirmed the aforementioned results (Figure 4(c)). Collectively, these in vitro experiments suggested that adropin may inhibit the calcification of VSMCs.

### 3.5. Adropin Inhibits STAT3 Entry into the Nucleus in Osteogenic Differentiated VSMCs In Vitro

To elucidate the inhibitory impact of adropin in the JAK2/STAT3 signaling pathway, entry of STAT3 into the nucleus was evaluated in each group of VSMCs. Results of the present study demonstrated that the protein expression levels of STAT3 in the nucleus were decreased in osteogenic differentiated VSMCs following adropin overexpression (Figures 5(a) and 5(b)). However, the protein expression levels of STAT3 in the cytoplasm did not exhibit any significant changes. Collectively, the results demonstrated that adropin inhibited entry of STAT3 into the nucleus in osteogenic differentiated VSMCs in vitro.

### 3.6. Adropin Inhibits Osteogenic Differentiation of VSMCs via the JAK2/STAT3 Signaling Pathway In Vitro

The role of the JAK2/STAT3 signaling pathway in osteogenic differentiation was investigated following modulation of the adropin expression. Notably, the results of the present study demonstrated that the mRNA expression levels of calcification-associated markers (BMP2, ALP, OPG, OCN, and Runx2) in VSMCs were decreased following adropin knockdown or treatment with AG490 (a JAK2 inhibitor; Figure 6(a)). Subsequently, the ALP activity of VSMCs was investigated, and results of the present study demonstrated that STAT3 knockdown or AG490 treatment also decreased the activity of ALP in vitro (Figure 6(b)). Additionally, the protein expression levels of calcification-associated markers (BMP2, ALP, OPG, OCN, and Runx2) were decreased following adropin knockdown in VSMCs and AG490 treatment (Figure 6(c)). These results indicated that adropin inhibited the osteogenic differentiation of VSMCs via the JAK2/STAT3 signaling pathway in vitro.

### 3.7. Adropin Alleviates Vascular Calcification In Vivo

Subsequently, whether adropin treatment also alleviated calcification in vivo was investigated. Compared with the control group, the protein expression levels of calcification-associated markers (ALP, OPG, OCN, smooth muscle protein 22 (SM22), Runx2, and *α*-smooth muscle actin (SMA)) in vascular tissues were significantly decreased following treatment with adropin (Figures 7(a) and 7(b)). This result was also confirmed using PCR analysis (Figure 7(c)). Moreover, the calcification-associated markers in rat vascular tissues and the osteogenic differentiation-associated markers in rat blood also exhibited significant reductions following adropin treatment (Tables 1 and 2). In summary, the results of the present study revealed that adropin inhibited vascular calcification in vivo.

## 4. Discussion

Vascular calcification is characterized by the deposition of hydroxyapatite mineral in the form of calcium-phosphate complexes in the vasculature [12]. At present, vascular calcification is regarded as a basis of a healthy aging process; however, it also plays a role in certain pathological processes, such as hypertension, chronic kidney disease, diabetes, and rare hereditary disorders [13, 14]. Numerous previous studies have demonstrated that vascular calcification is an actively and tightly regulated process, which is similar to that of bone development and cartilage formation [15]. The transdifferentiation of VSMCs into osteoblast-like cells is identified as a key event in the progression of vascular calcification [3, 4]. Therefore, the pathophysiological mechanisms that drive vascular calcification require further exploration, and the development of novel therapeutic options is required.

Adropin was initially identified in 2008, as a protein encoded by the energy homeostasis associated gene [16]. In recent years, adropin has been more widely researched due to its critical role in various cardiovascular diseases [7, 17]. Wang et al. demonstrated that adropin inhibited the phenotypic modulation and proliferation of VSMCs during neointimal hyperplasia via the AMPK/ACC axis [18]. However, the specific influence of adropin on the osteogenic differentiation of VSMCs remained to be fully elucidated. The results of the present study demonstrated that the expression of adropin was increased in calcific vascular tissues and osteogenic differentiated VSMCs. Moreover, results of the present study demonstrated that adropin alleviated vascular calcification in vivo. In addition, the results of the present study highlighted that adropin may inhibit the osteogenic differentiation of VSMCs via the JAK2/STAT3 axis in vitro. These results suggested that adropin may act as a potential therapeutic target for vascular calcification.

Our research also found that adropin was downregulated in in vivo and in vitro calcification models, which caught our interest, as some undetected mechanisms might regulate the content of adropin in cells or animal models. Some upstream of adropin had already been reported recently. For example, Li and Xie found that HDAC11-mediated histone deacetylation may inhibit the level of adropin to suppress atherosclerosis [19]. In the future, it is valuable to deeply explore the underlying mechanism of adropin treatment in vascular calcification, which may provide more evidences and targets for adropin treatment. Furthermore, we would also try to clarify the upstream to regulate the level of adropin in vascular tissues, for histone deacetylation, m6A methylation, and some other regulated mechanism. These upstream might be more meaningful for researchers to develop target inhibitors.

Previous studies reported that the JAK2/STAT3 axis regulated the cellular metabolism of VSMCs. For example, Han et al. demonstrated that cytokine-induced apoptosis inhibitor 1 accelerated the vascular remodeling of VSMCs via JAK2/STAT3 in vitro [20]. Hossain et al. also demonstrated that Ang II increased nitroxidative stress via the JAK2/STAT3 pathway, which may cause the overexpression of Gi*α* proteins and cell cycle-associated proteins, and the hyperproliferation of VSMCs [21]. Based on these experiments, the present study is aimed at further investigating whether the JAK2/STAT3 axis also participated in the process of VSMC calcification in vitro. The results of the present study revealed that adropin inhibited osteogenic differentiation of VSMCs via the JAK2/STAT3 signaling pathway in vitro. These findings provide a theoretical basis for the development of novel therapeutic regimes involving the JAK2/STAT3 axis in vascular calcification. As suggested by Wang et al., STAT3 may promote the transcription of target genes, such as adropin [22]. Wang et al. found that higher adropin levels in the blood are associated with STAT3 in diabetes [22]. STAT3 is involved in the genetic regulation of adropin, increasing the levels of circulating adropin and promoting Enho expression in the livers of diabetic rats [22]. For future studies, we could try to explore the role of JAK2/STAT3 axis in animal models and confirm whether the JAK2/STAT3 axis also shows its function of adropin treatment in vivo. Furthermore, it is essential to study if JAK2/STAT3 may also act as the downstream of some other mechanisms in the process of vascular calcification. These findings would support researchers to develop JAK2/STAT3 target inhibitor for vascular calcification treatment.

In conclusion, to the best of our knowledge, the present study was the first to demonstrate the specific therapeutic mechanism of adropin in vascular calcification. Notably, the results of the present study demonstrated that adropin alleviated vascular calcification in vivo. Moreover, adropin may also inhibit the osteogenic differentiation and calcification of VSMCs in vitro, and the JAK2/STAT3 signaling pathway may play a key role in this process. Thus, these findings may be beneficial for further elucidating the molecular mechanism associated with the protective effects of adropin in vascular calcification.

## Figures and Tables

**Figure 1:** Adropin is expressed at low levels in calcific vascular tissues and osteogenic differentiated VSMCs. (a, b) The protein expression of adropin in rat vascular tissues and VSMCs was quantified using western blotting. GAPDH was used as the loading control. (c) The mRNA expression levels of adropin in VSMCs were quantified using reverse-transcription quantitative PCR. GAPDH was used as the loading control. (d, e) The expression of adropin in VSMCs was evaluated using immunofluorescence. Each experiment was performed three times, and data are presented as the mean ± SD. VSMCs: vascular smooth muscle cells. ^#^*p* <0.05 compared to vehicle.

**Figure 2:** Adropin inhibits JAK2/STAT3 activation in osteogenic differentiated VSMCs in vitro. (a) The activation of the JAK2/STAT3 signaling pathway in VSMCs was quantified using western blotting. GAPDH was used as the loading control. (b) Reverse-transcription quantitative PCR was carried out to demonstrate the efficiency of adropin knockdown and overexpression in VSMCs. GAPDH was used as the loading control. (c) The phosphorylation of the JAK2/STAT3 signaling pathway in VSMCs. Each experiment was performed three times, and data are presented as the mean ± SD. JAK2: tyrosine protein kinase JAK2; STAT3: signal transducer and activator of transcription 3; VSMCs: vascular smooth muscle cells. ^∗^*p* < 0.05 compared to control. ^#^*p* < 0.05 compared to the Cacl_2_ group.

**Figure 3:** Adropin inhibits VSMC osteogenic differentiation in vitro. (a, b) The protein expression levels of calcification-associated markers (BMP2, ALP, OPG, OCN, and Runx2) in VSMCs were quantified using western blotting. GAPDH was used as the loading control. Each experiment was performed three times, and data are presented as the mean ± SD. VSMCs: vascular smooth muscle cells; BMP2: bone morphogenetic protein 2; ALP: alkaline phosphatase; OPG: osteoprotegerin; OCN: osteocalcin; Runx2: runt-related transcription factor 2. ^∗^*p* < 0.05 compared to control. ^#^*p* < 0.05 compared to the Cacl_2_ group.

**Figure 4:** Adropin inhibits VSMC calcification in vitro. (a) The calcification of VSMCs was evaluated using alizarin red staining. (b) The concentration of calcium ions in VSMCs was assessed. (c) The mRNA expression levels of calcification-associated markers (BMP2, ALP, OPG, OCN, and Runx2) in VSMCs were quantified using reverse-transcription quantitative PCR. GAPDH was used as the loading control. Each experiment was performed three times, and data are presented as the mean ± SD. VSMCs: vascular smooth muscle cells; BMP2: bone morphogenetic protein 2; ALP: alkaline phosphatase; OPG: osteoprotegerin; OCN: osteocalcin; Runx2: runt-related transcription factor 2. ^∗^*p* < 0.05 compared to control. ^#^*p* < 0.05 compared to the Cacl_2_ group.

**Figure 5:** Adropin inhibits STAT3 entry into the nucleus in osteogenic differentiated VSMCs in vitro. (a, b) The entry of STAT3 into the nucleus of VSMCs was evaluated using western blotting. GAPDH was used as the loading control. Each experiment was performed three times and data are presented as the mean ± SD. STAT3: signal transducer and activator of transcription 3; VSMCs: vascular smooth muscle cells. ^∗^*p* < 0.05 compared to control. ^#^*p* < 0.05 compared to the Cacl_2_ group.

**Figure 6:** Adropin inhibits osteogenic differentiation of VSMCs via the JAK2/STAT3 signaling pathway in vitro. (a) The mRNA expression levels of calcification-associated markers (BMP2, ALP, OPG, OCN, and Runx2) in VSMCs were quantified using reverse-transcription quantitative PCR. GAPDH was used as the loading control. (b) The ALP activity of VSMCs. GAPDH was used as the loading control. (c) The protein expression levels of calcification-associated markers (BMP2, ALP, OPG, OCN, and Runx2) in VSMCs were quantified using western blotting. GAPDH was used as the loading control. Each experiment was performed three times, and data are presented as the mean ± SD. VSMCs: vascular smooth muscle cells; JAK2: tyrosine protein kinase JAK2; STAT3: signal transducer and activator of transcription 3; BMP2: bone morphogenetic protein 2; ALP: alkaline phosphatase; OPG: osteoprotegerin; OCN: osteocalcin; Runx2: runt-related transcription factor 2. ^∗^*p* < 0.05 compared to control. ^#^*p* < 0.05 compared to the Cacl_2_ group.

**Figure 7:** Adropin alleviates vascular calcification in vivo. (a)–(c) The protein expression levels of calcification-associated markers (ALP, OPG, OCN, SM22, Runx2, and *α*-SMA) in rat vascular tissues were quantified using western blotting. GAPDH was used as the loading control. Each experiment was performed three times, and data are presented as the mean ± SD. ALP: alkaline phosphatase; OPG: osteoprotegerin; OCN: osteocalcin; SM22: smooth muscle protein 22; Runx2: runt-related transcription factor 2; *α*-SMA: *α*-smooth muscle actin. ^∗^*p* < 0.05 compared to control. ^#^*p* < 0.05 compared to the model+saline group.

**Table 1:** The characteristic of calcification in rats' aortas.

	Ca^2+^ (nmol/mg)	ALP (IU/g)
Control	11.22 ± 1.26	178.04 ± 31.25
Model+saline	62.54 ± 3.67	512.45 ± 45.79
Model+adropin	23.15 ± 2.41^∗^	264.15 ± 36.88^∗^

^∗^Significantly difference (comparing with the model+saline group).

**Table 2:** The characteristic of osteogenic differentiation in rats' blood.

	PTH (pg/ml)	BALP (pg/ml)	OC (ng/ml)	Ca (mmol/L)
Control	42.56 ± 3.64	623.54 ± 105.23	6.23 ± 0.38	2.11 ± 0.23
Model+saline	18.45 ± 2.45	785.64 ± 111.46	10.26 ± 0.64	1.01 ± 0.15
Model+adropin	33.45 ± 3.61^∗^	634.54 ± 104.56^∗^	6.89 ± 0.42^∗^	1.84 ± 0.26^∗^

^∗^Significantly difference (comparing with the model+saline group).

## Data Availability

The datasets used or analyzed during the current study are available from the corresponding author on reasonable request.

## Supplementary Materials

Supplementary Materials Supplementary Table S1: antibodies table. Supplementary Table S2: primers used for PCR.
